The article "Evaluation of ABC Bleeding Score and SAMe-TT2R2 Score on the Risk of Bleeding after Anticoagulation in Patients with Nonvalvular Atrial Fibrillation Complicated with Coronary Heart Disease" was retracted in 2023. Reasons: signs of a paper mill; compromised peer review; unreliable results or conclusions.

# Evaluation of ABC Bleeding Score and SAMe-TT2R2 Score on the Risk of Bleeding after Anticoagulation in Patients with Nonvalvular Atrial Fibrillation Complicated with Coronary Heart Disease

**DOI:** 10.1155/2022/6982753

**Published:** 2022-09-28

**Authors:** Meiling Du, Feixing Li, Aiai Zhang, Fangjiang Li, Xiaoyuan Wang

**Affiliations:** The First Affiliated Hospital of Hebei North University, Zhangjiakou 075400, Hebei, China

## Abstract

**Objective:**

To explore the predictive value of ABC bleeding score and SAMe-TT2R2 score on the risk of bleeding in patients with nonvalvular atrial fibrillation (NVAF) complicated with coronary heart disease (CHD) after anticoagulation.

**Methods:**

149 patients with NVAF complicated with CHD were followed up in our hospital for one year. The bleeding events during the follow-up period were observed, the ABC bleeding score and SAMe-TT2R2 score were calculated, the predictive value of the two scoring methods for the main bleeding risk was analyzed by the ROC curve, and the AUC area under the ROC curve of the two scoring methods was compared by the Delong test.

**Results:**

There were 32 bleeding events during the follow-up period. The AUC of ABC bleeding score and SAMe-TT2R2 score were 0.775 (*P* < 0.01) and 0.624 (*P* < 0.05), respectively. The Delong test showed that the AUC of ABC bleeding score was significantly higher than that of SAMe-TT2R2 score (*d* = 2.177, *P* < 0.05).

**Conclusion:**

Both the ABC bleeding score and SAMe-TT2R2 score can predict the risk of bleeding after anticoagulation in patients with NVAF and CHD. The critical value of the SAMe-TT2R2 score for predicting bleeding events in patients with NVAF and CHD may need to be increased to 4 or 5, and the prediction ability of ABC bleeding score is significantly better than that of the SAMe-TT2R2 score.

## 1. Introduction

Risk factors for nonvalvular atrial fibrillation and coronary heart disease are similar, such as age, alcohol consumption, and underlying medical conditions such as diabetes and hypertension. The clinical incidence of both the diseases is very high, and it is increasing year-by-year. Studies have shown that about 33% of patients with atrial fibrillation have coronary heart disease [1]. For the antithrombotic treatment of atrial fibrillation complicated with coronary heart disease, dual antiplatelet therapy (DAPT) is recommended to avoid stent thrombosis, and different oral anticoagulants (OAC) are reasonably selected. In this way, stroke and organ embolism can be prevented. However, antithrombotic therapy for both the diseases increases the risk of bleeding in patients. In order to weigh the risk of vascular embolism and bleeding, a large number of studies have discussed the choice of drugs and the setting of the course of antithrombotic therapy. However, choosing an appropriate individualized antithrombotic regimen is still a difficult clinical treatment [2–5]. At present, various scores are used to assess the bleeding risk after anticoagulation in patients with atrial fibrillation, but whether it is suitable for patients with atrial fibrillation and coronary heart disease is still inconclusive [6]. The SAMe-TT2R2 score was proposed by Apostolakis [7] in 2013, which is used to predict the anticoagulation efficacy of warfarin in patients with atrial fibrillation and provide a reference for the selection of anticoagulant drugs. The ABC bleeding score was proposed by Hijazi [8] and others in 2016, which combined clinical characteristics and biomarkers to assess the bleeding risk of patients with atrial fibrillation. This article aims to evaluate the predictive value of SAMe-TT2R2 score and ABC bleeding score for clinically significant bleeding events in patients with atrial fibrillation and coronary heart disease after the anticoagulation therapy.

The article "Evaluation of ABC Bleeding Score and SAMe-TT2R2 Score on the Risk of Bleeding after Anticoagulation in Patients with Nonvalvular Atrial Fibrillation Complicated with Coronary Heart Disease" was retracted in 2023. Reasons: signs of a paper mill; compromised peer review; unreliable results or conclusions.

## 2. Materials and Methods

### 2.1. Research Objects

Patients with nonvalvular atrial fibrillation and coronary heart disease who received anticoagulation therapy in our hospital from March 2018 to September 2020 and completed 1-year follow-up were selected as the research subjects. The inclusion criteria include the following: (1) meet the diagnostic criteria for nonvalvular atrial fibrillation; (2) the previous diagnosis of coronary atherosclerotic heart disease (a clear history of myocardial infarction or imaging evidence of coronary artery disease); (3) agree to participate in this study and sign the informed consent. The exclusion criteria include the following: ⑴ those with heart valve disease. (2) those with active bleeding, clinically significant bleeding or abnormal coagulation function, and other prone to bleeding constitution; (3) those with a history of peptic ulcer disease; (4) patients whose hypertension has not achieved satisfactory control effect; (5)patients with active malignant tumor disease or those whose expected survival time is limited to less than 12 months due to severe diseases. According to the above criteria, a total of 149 subjects were included in this study. There were 78 males and 71 females, aged 55–77 years, with a median age of 67 (63–70) years. There were 57 cases of smoking and 133 cases of 3 underlying diseases (hypertension, diabetes, coronary atherosclerotic heart disease, congestive heart failure, chronic lung disease, stroke, peripheral vascular disease, liver disease, and kidney disease). There were 93 cases of hypertension, 71 cases of heart failure, and 40 cases of diabetes. Forty-five patients were treated with warfarin anticoagulation, and 103 patients were treated with antiplatelet drugs. Among them, 9 patients received anticoagulation combined with the antiplatelet therapy, and 10 patients did not receive the antithrombotic therapy. This study was reviewed and approved by the Institutional Ethics Review Board of the First Affiliated Hospital of Hebei North University.

The article "Evaluation of ABC Bleeding Score and SAMe-TT2R2 Score on the Risk of Bleeding after Anticoagulation in Patients with Nonvalvular Atrial Fibrillation Complicated with Coronary Heart Disease" was retracted in 2023. Reasons: signs of a paper mill; compromised peer review; unreliable results or conclusions.

### 2.2. Research Methods and Bleeding Risk Score

The ABC bleeding score and the SAMe-TT2R2 score were both performed by two doctors, and if there was any inconsistency, they were checked and confirmed by a third person. The ABC bleeding score refers to the method proposed by Hijazi et al. [8]. The patient's clinical characteristics (age and bleeding history) and biomarkers (cystatin C, troponin T (TnT), and hemoglobin), a total of 5 factors, were entered into the ABC bleeding score calculation table, and the score was calculated. The corresponding risk value was obtained by matching the score with the bleeding risk. A 1-year bleeding risk of <1% is defined as low risk, 1% to 2% as intermediate risk, and >2% as high risk. The SAMe-TT2R2 score refers to the method proposed by Apostolakis et al. [7], including 1 point for women, 1 point for age <60 years, and 1 point for 3 underlying diseases. The use of drugs that interact with warfarin during treatment (digoxin, amiodarone, *β*-blockers, calcium antagonists, ARB/ACEIs, statins, and hypoglycemic agents) is for 1 point, 2 points for smoking history within 2 years, and 2 points for race (nonwhite). There are a total of 6 items, and the score is calculated, with a maximum score of 8 points.

### 2.3. Evaluation and Collection of Clinically Significant Bleeding Events

The clinically significant bleeding events in this study were defined as clinically obvious signs of bleeding (including imaging) accompanied by a decrease in hemoglobin of 2 g/dL or more or a decrease in hematocrit by more than 9% compared with the initial screening, transfusion of 2 or more units of red blood cells or whole blood. If fatal or bleeding from a critical site or organ (intracranial, intraspinal, intraocular, pericardial, intraarticular, retroperitoneal, or intramuscular with compartment syndrome), bleeding events requiring clinical treatment (endovascular tamponade, endoscopic hemostasis, interventional embolization, puncture and drainage, surgery, reduction/discontinuation of antiplatelet, and anticoagulant drugs). Major bleeding events were collected based on the patient's hospitalization data, outpatient follow-up, and telephone follow-up.

The article "Evaluation of ABC Bleeding Score and SAMe-TT2R2 Score on the Risk of Bleeding after Anticoagulation in Patients with Nonvalvular Atrial Fibrillation Complicated with Coronary Heart Disease" was retracted in 2023. Reasons: signs of a paper mill; compromised peer review; unreliable results or conclusions.

### 2.4. Statistical Methods

The data were processed and analyzed by SPSS 25.0 software, the measurement data were expressed as (`*x* ± *s*), the count data were expressed as rate (%), and the ROC curve was drawn by SPSS software. The Delong test was used to compare the AUC area under the ROC curve of the two scoring methods, and *P* < 0.05 was considered to be statistically significant.

## 3. Results

### 3.1. Distribution of Patients under the Two Scores

In the ABC bleeding score, 5 cases were in the low-risk group, 83 in the intermediate-risk group, and 61 in the high-risk group. In the SAMe-TT2R2 score, the lowest score was 2 points, including 24 cases with £3 points, 46 cases with 4 points, 53 cases with 5 points, and 26 cases with ³6 points. In the ABC bleeding score, there was no significant difference in the rates of anticoagulation, antiplatelet and no antithrombotic therapy among the low, medium, and high-risk groups (*P* > 0.05). In the SAMe-TT2R2 score, there was no significant difference in the anticoagulation, antiplatelet, and no antithrombotic treatment rates between the £3, 4, 5, and ³6 groups (*P* > 0.05), as shown in Table 1.

### 3.2. Influencing Factors and Score Comparison of Bleeding Events

As shown in Table 2, patients with nonvalvular atrial fibrillation and coronary heart disease were divided into two groups according to whether they were bleeding or not, and then the general data, bleeding risk factors, and scores were compared between the two groups. There was no significant difference in gender, age, smoking, hypertension, diabetes, and heart failure between the two groups (*P* > 0.05). There was a statistically significant difference in the proportion of previous bleeding history (*P* < 0.01). There were significant differences in the SAMe-TT2R2 score and ABC bleeding score (*P* < 0.01).

### 3.3. Score Results and Occurrence of Bleeding Events

Followed up for 1 year, there were 32 cases (21.5%) of total bleeding. In the ABC bleeding score, there was a statistically significant difference in the incidence of total bleeding events between the low, medium, and high-risk groups (*c*^*2*^ = 22.377, *P* < 0.01). There was a statistically significant difference in the incidence of bleeding events between the low-intermediate risk group (*n* = 88) and the high-risk group (*c*^*2*^ = 23.305, *P* < 0.01). There was a statistically significant difference in the incidence of bleeding events between the intermediate-risk group and the high-risk group (*c*^2^ = 21.553, *P* < 0.01). There was no significant difference in the incidence of bleeding events between the £3, 4, 5, and ³6 groups in the SAMe-TT2R2 score (*c*2 = 5.170, *P*=0.160), as shown in Table 3.

The article "Evaluation of ABC Bleeding Score and SAMe-TT2R2 Score on the Risk of Bleeding after Anticoagulation in Patients with Nonvalvular Atrial Fibrillation Complicated with Coronary Heart Disease" was retracted in 2023. Reasons: signs of a paper mill; compromised peer review; unreliable results or conclusions.

### 3.4. Comparison of Predictive Ability of ABC Bleeding Score and SAMe-TT2R2 Score

SPSS software was used to draw the ROC curve of ABC bleeding score and SAMe-TT2R2 score to evaluate the bleeding risk of patients within 1 year, and the AUC was compared. The AUC of SAMe-TT2R2 score was 0.624 (*P* < 0.05, 95% *CI*: 0.515–0.734), the Youden index was 0.200, and the corresponding threshold was 4.5 points. The ABC bleeding score AUC was 0.775 (*P* < 0.01, 95% *CI*: 0.695–0.855), the Youden index was 0.510, and the corresponding threshold was 12.75 points. Furthermore, the Delong test showed that there was a statistically significant difference in AUC under the ROC curve between the two scoring methods (*D* = 2.177, *P* < 0.05, 95% CI: 0.015–0.287), see in Figure 1.

## 4. Discussion

Coronary heart disease and atrial fibrillation are considered to be the most common clinical cardiovascular diseases. The prevalence of the two diseases increased significantly with age, and there were similar high-risk factors, and there was also a certain relationship between atrial fibrillation and coronary heart disease. Patients with coronary heart disease have coronary multivessel disease, sinoatrial node or atrioventricular node branch disease, myocardial infarction (especially large myocardial infarction), and atrial myocardial ischemia. Atrial fibrillation is more likely to occur when combined with mitral regurgitation, heart failure, and hypertension. The possible mechanism is that the above conditions lead to increased left atrial load and left atrial dilation, thereby increasing the incidence of atrial fibrillation in patients with coronary heart disease [9]. The incidence of atrial fibrillation in ³65-year-old patients with acute myocardial infarction was as high as 22.1% [10]. Coronary heart disease patients with atrial fibrillation need to be combined with DAPT on the basis of OAC antithrombotic therapy after PCI, which increases the risk of bleeding by 2–3 times. For these patients, it is recommended to use a scoring tool to minimize the duration of triple antithrombotic therapy. And according to the severity of coronary artery disease in patients, the drug compatibility is reasonably selected to optimize the antithrombotic treatment [11], so as to reduce the occurrence of bleeding events while conducting effective antithrombotic treatment. Therefore, it is necessary to choose a more reasonable bleeding score to predict bleeding risk.

Currently, both the SAMe-TT2R2 score and the ABC bleeding score can be used to assess the bleeding risk after anticoagulation in patients with atrial fibrillation. However, there is no comparison on the predictive value of bleeding risk in Chinese patients with atrial fibrillation complicated by coronary heart disease. Therefore, this paper explores and compares the predictive value of SAMe-TT2R2 score and ABC bleeding score for clinically significant bleeding events in patients with atrial fibrillation and coronary heart disease. The results showed that both the methods could predict the bleeding risk of patients, and the predictive effect of the ABC bleeding score was significantly better than that of the SAMe-TT2R2 score. Studies have shown that the higher the SAMe-TT2R2 score of patients, the greater the risk of adverse reactions [12, 13]. The SAMe-TT2R2 score assignment is influenced by race, with the main studies focusing on nonwhite populations [14–16]. The lowest score of patients in my country is 2 points, so there will be a phenomenon of high SAMe-TT2R2 score. Its adaptability in the nonwhite population needs to be confirmed by large-scale population studies. Some studies have suggested that the use of SAMe-TT2R2 score to predict the risk of bleeding in Chinese may need to increase the threshold to 4 or 5. The study population consisted of patients with atrial fibrillation and coronary heart disease, combining the risk factors of the two diseases, especially the characteristic that the incidence rate increases with age. The total SAMe-TT2R2 score was high in this study, and the corresponding threshold of the ROC curve of the obtained SAMe-TT2R2 score was 4.5 points. Currently, doctors around the world prefer to use nonvitamin K oral anticoagulants, namely new oral anticoagulants (NOACs) [17]. At the same time, some high bleeding risk parameters and elevated serum creatinine values were independent predictors of oral anticoagulant choice, resulting in inconsistency with the prediction results of the SAMe-TT2R2 score. It is suggested that some basic bleeding risk factors may need to be added to improve the predictive discrimination ability of the SAMe-TT2R2 score.

The article "Evaluation of ABC Bleeding Score and SAMe-TT2R2 Score on the Risk of Bleeding after Anticoagulation in Patients with Nonvalvular Atrial Fibrillation Complicated with Coronary Heart Disease" was retracted in 2023. Reasons: signs of a paper mill; compromised peer review; unreliable results or conclusions.

Based on age, previous bleeding history, and three biomarkers (hemoglobin, cTn-hs, and GDF-15 or cystatin C), the ABC bleeding score more comprehensively incorporates the influencing factors of patients' bleeding, compared with the SAMe-TT2R2 score. Compared with the SAMe-TT2R2 score, the ABC bleeding score more comprehensively incorporates the influencing factors of patients' bleeding. The addition of biomarkers to predictive models attenuated the predictive importance of many clinical variables (e.g., diabetes mellitus and previous stroke). The ABC bleeding score includes biomarkers that may indicate underlying bleeding-related organ dysfunction in these diseases, and thus some clinical variables have no effect on the prognosis of major bleeding. Related studies were validated in a large cohort of patients with atrial fibrillation receiving anticoagulation, and the ABC bleeding score was superior to the HAS-BLED and ORBIT scores as a decision support for anticoagulation in patients with atrial fibrillation. It performed equally well in subgroups of patients receiving the antiplatelet therapy and different anticoagulant therapy [8, 18, 19] to achieve an optimal balance between stroke risk reduction and associated bleeding risk for each patient. Compared to models based solely on clinical data and routine laboratory testing, the ABC bleeding score introduces a panel of biomarkers that may be indicative of tissue fragility, organ dysfunction, and clinically unrecognized disease. This provides better targeting and fewer overlapping risk factors, providing a more robust tool for risk stratification and further optimizing anticoagulant treatment decisions in patients with AF.

In conclusion, both SAMe-TT2R2 score and ABC bleeding score can predict the bleeding risk after anticoagulation in patients with atrial fibrillation and coronary heart disease. The critical value of SAMe-TT2R2 score for predicting bleeding events in atrial fibrillation complicated with coronary heart disease may need to be increased to 4 or 5, and the predictive ability of ABC bleeding score is significantly better than that of the SAMe-TT2R2 score. Combined with the predicted results of the ABC bleeding score, the anticoagulation therapy for patients with atrial fibrillation and coronary heart disease is more required to be individualized, and the optimal drug regimen suitable for the patient should be selected to prevent stroke and embolic events and reduce the risk of bleeding.

## Figures and Tables

**Figure 1:** ROC curve comparison of the ABC bleeding score and SAMe-TT2R2 score.

**Table 1:** The risk stratification distribution of two different scores (number of cases (%)).

Antithrombotic therapy	ABC bleeding score				SAMe-TT2R2 score				
	Low-risk group (5 cases)	Intermediate risk group (83 cases)	High-risk group (61 cases)	*P* value	£3 points (24 cases)	4 points (46 cases)	5 points (53 cases)	³6 points (26 cases)	*P* Value
Anticoagulant therapy	2 (40.0)	25 (30.1)	18 (29.5)	0.886	5 (20.8)	13 (28.3)	14 (26.4)	13 (50.0)	0.099
Antiplatelet therapy	2 (40.0)	57 (68.7)	44 (72.1)	0.303	19 (79.2)	30 (65.2)	37 (69.8)	17 (65.4)	0.649
Nonantithrombotic therapy	1 (20.0)	5 (6.0)	4 (6.6)	0.431	1 (4.2)	4 (8.7)	4 (7.5)	1 (3.8)	0.910

**Table 2:** Comparison of general data, risk factors, and scores between the two groups of patients.

Projects	No new bleeding (*n* = 117)	New bleeding (*n* = 32)	*t*/*c*^*2*^/*Z*	*P* value
Female cases (%)	55 (47.0)	16 (50.0)	0.09	0.764
Age (y)	67 ± 5	68 ± 5	0.829	0.408
Smoking cases (%)	42 (35.9)	15 (46.9)	1.282	0.258
Past bleeding cases (%)	10 (8.5)	10 (31.3)	9.277	0.002
High blood pressure cases (%)	74 (63.2)	19 (59.4)	0.161	0.689
Diabetes cases (%)	29 (24.8)	11 (34.4)	1.176	0.278
Heart failure cases (%)	52 (44.4)	19 (59.4)	2.246	0.134
SAMe-TT2R2 score	4.5 ± 1.0	5.0 ± 1.0	2.246	0.025
ABC bleeding score	12.5 ± 2.4	14.8 ± 1.5	4.774	0.000

The article "Evaluation of ABC Bleeding Score and SAMe-TT2R2 Score on the Risk of Bleeding after Anticoagulation in Patients with Nonvalvular Atrial Fibrillation Complicated with Coronary Heart Disease" was retracted in 2023. Reasons: signs of a paper mill; compromised peer review; unreliable results or conclusions.

**Table 3:** Comparison of bleeding events in two different stratification scores (number of cases (%)).

	ABC bleeding score				SAMe-TT2R2 score				
	Low-risk group (5 cases)	Intermediate risk group (83 cases)	High-risk group (61 cases)	*P* value	£3 points (24 cases)	4 points (46 cases)	5 points (53 cases)	³6 points (26 cases)	*P* value
Total bleeding events	0	7 (8.4)	25 (41.0)	0.000	3 (12.5)	7 (15.2)	13 (24.5)	9 (34.6)	0.160
Intracerebral hemorrhage	0	0	2 (3.3)		0	0	1 (1.9)	1 (3.8)	
Gastrointestinal bleeding	0	4 (4.8)	13 (21.3)		1 (4.2)	5 (10.9)	7 (13.2)	4 (15.4)	
Other bleeding	0	3 (3.6)	10 (16.4)		2 (8.3)	2 (4.3)	5 (9.4)	4 (15.4)	

## Data Availability

The data that support the findings of this study are available from the corresponding author upon reasonable request.
